# Stable Median Centre Clustering for Unsupervised Domain Adaptation Person Re-Identification

**DOI:** 10.1155/2021/2883559

**Published:** 2021-07-21

**Authors:** Jifeng Guo, Wenbo Sun, Zhiqi Pang, Yuxiao Fei, Yu Chen

**Affiliations:** College of Information and Computer Engineering, Northeast Forestry University, Harbin 150040, China

## Abstract

The current unsupervised domain adaptation person re-identification (re-ID) method aims to solve the domain shift problem and applies prior knowledge learned from labelled data in the source domain to unlabelled data in the target domain for person re-ID. At present, the unsupervised domain adaptation person re-ID method based on pseudolabels has obtained state-of-the-art performance. This method obtains pseudolabels via a clustering algorithm and uses these pseudolabels to optimize a CNN model. Although it achieves optimal performance, the model cannot be further optimized due to the existence of noisy labels in the clustering process. In this paper, we propose a stable median centre clustering (SMCC) for the unsupervised domain adaptation person re-ID method. SMCC adaptively mines credible samples for optimization purposes and reduces the impact of label noise and outliers on training to improve the performance of the resulting model. In particular, we use the intracluster distance confidence measure of the sample and its *K*-reciprocal nearest neighbour cluster proportion in the clustering process to select credible samples and assign different weights according to the intracluster sample distance confidence of samples to measure the distances between different clusters, thereby making the clustering results more robust. The experiments show that our SMCC method can select credible and stable samples for training and improve performance of the unsupervised domain adaptation model. Our code is available at https://github.com/sunburst792/SMCC-method/tree/master.

## 1. Introduction

Person re-identification (re-ID) is an image retrieval task based on a given image of a person to identify the person in other images captured by different cameras [1, 2]. At present, person re-ID is widely used in the field of social security. Although research on person re-ID in a single domain has achieved satisfactory performance [3–5], manual annotation costs considerable manpower and material resources, and it is impractical to manually label new large-scale datasets [6]. Therefore, unsupervised person re-ID is proposed to solve the problem of the high-cost manual annotation, as it does not need labelled data, and thus, unnecessary costs are reduced. It is widely used on easily available unlabelled datasets and applied to practical scenes [7].

Unsupervised person re-ID lacks labelled data for supervision information [8, 9]. Moreover, cross-domain person re-ID has a domain shift problem caused by the differences in the fields of view, resolutions, and light occlusion levels among different domains, which result in a large performance drop for a model that performs well in the source domain when applied to the target domain [10–13]. Therefore, an unsupervised domain adaptation (UDA) method is proposed to solve the problem of domain shift in different feature spaces. The UDA method combines the given source domain data and target domain data to solve the problem of domain shift between different domains so that the model trained on the labelled data in the source domain can be adapted to unlabelled data in the target domain [14–17]. Among the different UDA methods, the method based on clustering to obtain pseudolabels to optimize the model has obtained the most advanced performance. This approach can be roughly divided into three steps: (1) pretraining the model with labelled data in the source domain; (2) performing feature extraction on the unlabelled data in the target domain with the pretrained model; (3) clustering the feature vector and fine-tuning the model according to the pseudolabels obtained by clustering [18]. Since this method relies on clustering to assign the same pseudolabel to samples belonging to the same cluster and then optimizes the model with the pseudolabel as the supervision information [19], the credibility of the pseudolabel determines the performance of the model [20]. If we have a highly credible pseudolabel, the model can be adapted to the target domain data [21–23]. However, in the original dataset, there may be some samples with label noise, and the noisy samples interfere with the model training process because of their incorrect information in the feature space. Therefore, only by selecting credible samples can we reduce the amplification of label noise during the training process and effectively apply to person re-ID tasks in different datasets.

To solve these problems, we propose a stable median centre clustering (SMCC) method to reduce the damage caused by potential label noise to the model and then obtain more stable clustering results to ensure the accuracy of pseudolabel assignment. Our SMCC method consists of two parts: a new reliable sample selection method and a new method for measuring the distances between clusters. First, instead of calculating distances from the centre point of the cluster to select credible samples, the SMCC method is more stable when there are many outliers in the feature space. By calculating the sum of the distances between the given sample and all other samples in the cluster, the offset of the median centre selected is smaller than the average centre point when there are outliers, which can better reflect the characteristics of the cluster. Furthermore, we select qualified credible sample points by calculating the distances between the current sample point and all other sample points in the cluster and the cluster proportion between the current sample point and its *K*-reciprocal nearest neighbour samples.

Figure 1 shows the iterative model adjustment process with credible sample selection. With the continuous optimization of the model, the samples belonging to the same cluster in the feature space become closer, and an increasing number of credible samples are selected. When the maximum number of iterations is reached, the samples belonging to the same cluster are clustered into the same cluster. We only select samples with high confidence in the early stage, and we reduce the misleading label noise during training to avoid the further amplification of label noise; thus, the performance of the model is improved to a certain extent. Second, compared with the previous intercluster distance calculation approach in which all sample points are equally valued, which leads to the damage of incorrect pseudolabel samples to intercluster distance, we obtain a credibility ranking list according to the intracluster distance among the samples and assign different weights to them according to the reliability of different sample points, which is the distance measurement between different clusters. For sample points with high confidence, we assign high weights to them, and we assign small weights to the sample points with low confidence that is still greater than the confidence threshold so that the model can take all credible samples into consideration and pay more attention to the feature information provided by the samples with high confidence.

Our contributions are summarized as follows. (1) We propose a stable median centre clustering (SMCC) method for unsupervised domain adaptation person re-ID, which uses the intracluster distances of samples and the cluster proportion of the *K*-reciprocal nearest samples as the criteria for obtaining credible samples. (2) We design a credibility ranking list for the samples in a cluster according to the intracluster distance and assign different weights to the sample points according to the ranking order for intercluster distance calculation. (3) Our experiments prove the superiority of our SMCC method, which achieves state-of-the-art performance on two popular person re-ID datasets, Market-1501 [24] and DukeMTMC-ReID [25, 26].

## 2. Related Work

### 2.1. Unsupervised Person Re-ID

With the development of deep learning, the existing person re-ID methods use convolutional neural networks for feature extraction and person retrieval [27–31]. In recent years, supervised person re-ID has been extensively studied and has achieved great performance [2, 32]. However, due to the large amount of overhead caused by manual labelling of large-scale datasets and because most of the data in practical applications are unlabelled data, researchers have begun to focus on studying unsupervised person re-ID. Different from supervised person re-ID, unsupervised person re-ID lacks labelled data as supervision information, which reduces the large cost of manual labelling. Unsupervised person re-ID can be widely used on easily available unlabelled datasets, which has great significance for practical applications. Different domains do not share the same feature space [33–36]; that is, there are large gaps in the resolution, background, lighting, and field of view of the original image in different domains, resulting in the problem of domain shift, which makes the effect of cross-domain person re-ID not ideal. Recently, an unsupervised person re-ID method based on cross-domain transfer learning was proposed to improve the performance of the resulting model on the unlabelled target domain with the labelled domain. Wang et al. proposed the TJ-AIDL method to learn attributes from the source domain and transfer them to the feature representation space of the target domain [10]. Zhao et al. [23] proposed a collaborative clustering and mutual instance selection method to enhance the performance of a cross-domain person re-ID model. Ge et al. [37] introduced a teacher-student model into an unsupervised person re-ID method and achieved satisfactory performance by refining the labels. Although unsupervised domain adaptation can solve the cross-domain shift problem, the source domain and the target domain do not share the same person identity in the re-ID problem, and the unsupervised domain adaptation method cannot be directly applied to the re-ID task effectively. Therefore, unsupervised domain adaptation re-ID is a challenging task at present.

### 2.2. Unsupervised Domain Adaptation Person Re-ID

The unsupervised domain adaptation (UDA) method was proposed to apply prior knowledge acquired from the source domain to an unlabelled target domain to reduce the impact of domain shift [7, 38, 39]. The current UDA methods can be roughly divided into three categories: GAN-based style transfer methods, feature information alignment methods between the source domain and target domain, and pseudolabel prediction methods used to explore the feature distributions of the unlabelled target domains. The first type of method mainly solves the problem of domain shift by narrowing the style difference between the source domain and the target domain. With a generative adversarial network, a labelled source domain image is transferred to an image with a style similar to the target domain style, and then, labelled data regarding the target domain style are obtained [40, 41]. These images are regarded as training samples for the model to adapt to the target domain [42, 43]. The second type of method aligns the feature information of different domains to obtain a domain-invariant feature space, thus reducing the influence of domain shifts between different domains [44, 45]. The third method involves clustering the unlabelled target domain data to explore the spatial distribution of the feature representation. It uses a pretrained model in the source domain to extract features in the target domain, performs a clustering algorithm on the obtained feature vectors, assigns the same pseudolabels to samples belonging to the same cluster, and then uses the pseudolabels as supervision information to fine-tune the model [46–49].

#### 2.2.1. GAN-Based Methods

In a previous study, Wei et al. [50] proposed a person transfer generative adversarial network (PTGAN), in which person images with labels were transferred to other unlabelled domains with a style transfer method to reduce the impact of domain shift. Similarly, on the basis of CycleGAN, SPAGN [51] was proposed with self-similarity and domain dissimilarity to avoid the loss of identity information from the generated image. To obtain a style transfer image similar to those of the target domain, Chen et al. proposed instance-guided context rendering to obtain a richer transfer image by transferring a person identity in the source domain to the context of the target domain [52].

#### 2.2.2. Feature Alignment Methods

To alleviate the view inconsistency between different domains, Yu et al. carried out asymmetric metric feature mapping for images in the source domain and target domain and mapped them to the same feature space in different ways for learning [17]. Wu et al. proposed a priori knowledge for learning cross-camera differences from the source domain to solve the domain shift caused by different camera views under the target domain and a camera-aware similarity consistency loss to learn cross-domain and cross-camera uniform pair similarity distributions [16]. Zhong et al. adjusted the gaps between the feature distributions of the source domain and target domain from the three perspectives of exemplar invariance, camera invariance, and neighbourhood invariance and fully explored the differences between cross-domain samples [53].

#### 2.2.3. Pseudolabel Prediction Methods

As an early clustering-based method, PUL [12] proposed by Fan et al. selects trusted samples to fine-tune the model by calculating the distances between sample points and cluster centre points. To mine the distinctive information contained in samples, Yang et al. proposed using PatchNet to generate multiple subimages for an input image and used global features and local features together for person re-ID [54]. Similarly, Fu et al. proposed dividing an image into a whole image, an upper part of the image, and a lower part of the image and performed clustering on these three parts to seek the potential similarities among the different parts [55]. The AD-Cluster [46] method generates style transfer images under different cameras with a GAN to increase the diversity of samples so that the performance of the resulting model is gradually improved throughout the adversarial learning process involving an image generator and a feature encoder. The PAST [20] method proposed by Zhang et al. divides the model training process into a conservative stage and a promoting stage to reduce the influence of label noise on the model through continuous iteration.

Although pseudolabel prediction methods perform better than the GAN-based methods and the feature alignment methods due to their examination of the spatial distribution of unlabelled samples, pseudolabel prediction methods cannot be further improved due to the influence of label noise in the dataset on clustering. If we select credible samples for training and avoid the amplification of label noise during the training process, a more reliable model can be obtained. The SMCC method takes the sample intracluster distance confidence (IDC) and the *K*-reciprocal nearest neighbour cluster proportion (KCP) as the sample credibility evaluation criteria and adds the samples that meet these criteria into the credible dataset during each iterative training process. Finally, a reliable pseudolabel dataset is obtained for model optimization to avoid the influence of noisy labels on the model.

## 3. Proposed Method

For UDA re-ID, we have a given label dataset {*X*_*S*_, *Y*_*S*_}, which contains *N*_*S*_ identities with *P*_*S*_ person images, where each *X*_*S*_^*i*^ corresponds to a unique identity label *Y*_*S*_^*i*^. Similarly, the unlabelled target domain dataset {*X*_*t*_} is also given, which contains *N*_*t*_ person images, but their labels *Y*_*t*_ are unknown. The purpose of our SMCC method is to explore the potential similarities between different samples in the target domain by clustering and combining the data of the labelled source domain and unlabelled target domain. Next, we expand on the SMCC method in further detail.

### 3.1. Overview

The overall framework of our proposed SMCC method is shown in Figure 2. The SMCC method first uses the style transfer model to obtain images, which are regarded as the pretraining data that are used to obtain a pretrained model that can adapt to the target domain. Then, clustering is performed on the unlabelled data in the target domain, and the sample points with higher confidence are selected according to the clustering results to ensure the pseudolabel correctness of the selected samples; thus, the influence of noisy samples on the model is reduced. Moreover, all the sample points are considered during the process of cluster merging, and different weights are assigned according to the obtained confidence degrees; this process ensures the full exploration of the feature spatial distribution and focuses on mining the potential differentiated information from the credible sample points. With the continuous optimization of the feature space, the number of credible samples gradually increases, and an increasing number of credible samples are used to fine-tune the CNN model to improve its robustness. In each clustering operation, when there is outlier interference, the offset of the median centre is smaller and is not affected as easily as the average centre; thus, the credible samples selected by our SMCC method avoid the inclusion of false pseudolabels.

### 3.2. Intracluster Distance Credibility Measurement

During the process of clustering, the sample points with higher similarity tend to belong to the same cluster; however, sample points belonging to the same cluster may be at the edge of the cluster. These points may belong to the current cluster or other clusters. To solve this problem, we propose an intracluster distance confidence (IDC) metric, which calculates the sum of the Euclidean distances from the current samples to all other sample points in the cluster, as the selection criterion for credible samples. We find that the total intracluster distance of the sample closest to the median cluster centre must be the smallest; that is, if the intracluster distance of a sample is smaller than that of the whole cluster, then it must be located near the median centre of the cluster, while if the intracluster distance of a sample is larger than that of the whole cluster, then it must be located at the edge of the cluster. The calculation formula of the sample intracluster distance is as follows:

(1) $$\begin{array}{c} D_{\text{ai}}=\sum_{j\in C_{a},j\neq i}E\left(C_{\text{ai}},C_{\text{aj}}\right), \end{array}$$

where *E*() represents the Euclidean distance between two samples, *C*_*a*_ represents all sample points in cluster *A*, and *C*_ai_ and *C*_aj_ represent a certain point and other different sample points in cluster *A*, respectively, and the sum of the Euclidean distances between a certain point and all other sample points in this cluster is calculated. Compared with the cluster centre points obtained by averaging all the feature vectors in the cluster, the points selected by our SMCC method are near the median centre of the cluster based on the sample's IDC, and the median centre points of the cluster are not greatly offset as the cluster centre points by the interference of outliers. The median centre point of a cluster is highly stable and reflects the central characteristics of the cluster [58]. It is worth noting that we do not directly calculate and sort the distances from the different sample points to the median centre of each cluster, but rather calculate the sum of the distances from each sample point to all other sample points in the cluster one by one because the distances obtained by the latter method are more accurate and better reflect the position information of the samples in the feature space. With this characteristic, we can take the IDC as the measurement criterion and select a sample located in the median centre of the cluster. Different from selecting a fixed distance as the threshold, we consider that the spatial distributions of different clusters may be different, so there is no excellent general distance threshold suitable for all clusters. Therefore, we calculate the intracluster distances of all samples in each cluster, establish a ranking list of intracluster distances from small to large, and select the first *M* samples from the ranking list as credible samples. In this way, we finally obtain the number of clusters multiplied by *M* credible samples for model training.

### 3.3. *K*-Reciprocal Nearest Neighbour Cluster Proportion

In addition to taking the IDC of each sample as the credible sample measurement criterion, we also take the spatial distribution of the *K*-reciprocal nearest neighbour samples of the current sample as another credible sample measurement criterion. The *K*-reciprocal nearest neighbour list of a sample can reflect the potential similarities of other samples near the current sample and accurately judge the confidence of the corresponding pseudolabels. Therefore, we propose the *K*-reciprocal nearest neighbour cluster proportion (KCP) to determine whether a given sample is credible. The equation for the KCP is as follows:

(2) $$\begin{array}{c} R_{\text{KCP}}\left(\chi_{t}\right)=\frac{\sum_{\chi_{i}\in K\left(\chi_{t}\right)}\alpha_{i}}{K}, \end{array}$$

where *K* is the number of samples that are the *K*-reciprocal nearest neighbour of sample *χ*_*t*_,

(3) $$\begin{array}{c} \alpha_{i}=\left\{\begin{array}{cc} 1, & \chi_{t}\text{ and }\chi_{i}\in C_{t},\\ 0, & \text{otherwise,} \end{array}\right) \end{array}$$

where *α*_*i*_ is the number of sample points in *K*-reciprocal nearest neighbour list *K*(*χ*_*t*_) that belong to the same cluster as the current sample point, and *R*_KCP_(*χ*_*t*_) ∈ [0, 1]. We find that the KCP can reflect the neighbourhood information of a sample near the current sample and judge whether the pseudolabel obtained by clustering is accurate. We regard samples larger than the KCP threshold as credible training samples; we regard samples less than the KCP threshold as unreliable samples. Finally, we select credible training samples according to the IDC and KCP measurement criteria.

### 3.4. Intercluster Distance Measurement

We not only propose the IDC credibility measurement but also propose a new measurement of intercluster distance, that is, according to the degree of the IDC within the same cluster, a dynamically weighted intercluster distance is established and is defined in the following formula:

(4) $$\begin{array}{c} D_{ab}=\frac{1}{n_{a}n_{b}}\sum_{i\in C_{a},j\in C_{b}}\partial_{ij}E\left(C_{a_{i}},C_{b_{j}}\right), \end{array}$$

where *n*_*a*_ and *n*_*b*_ represent the numbers of samples in cluster *A* and cluster *B*, respectively, *C*_*a*_ and *C*_*b*_ represent clusters *A* and *B*, respectively, and ∂_*ij*_ is the dynamic weight where its value is determined by the positions of the two samples in the intercluster distance ranking list. For samples with higher confidence at the top of the ranking list, we assign larger weights; in contrast, for samples with lower confidence at the bottom of the ranking list, we assign smaller weights. Equation (4) fully considers all the sample points from the two clusters in the clustering process, but for the samples with lower confidence, we reduce their contribution to the distance measurement. The dynamic weighting method can fully explore the spatial information of all samples during cluster merging, focus more on the valid information of credible samples, reduce false label noise that misleads the clustering results, and make the clustering results more accurate. The batch hard triplet loss and softmax cross-entropy loss are used in the loss function for source domain pretraining, and batch hard triple loss is used in the target domain, where the softmax cross-entropy loss is defined as follows:

(5) $$\begin{array}{c} L_{\text{soft max}}=-\sum_{i=1}^{P}\sum_{a=1}^{K}\log\frac{e^{W_{y_{a,i}}^{T}\chi_{a,i}}}{\sum_{K=1}^{C}e^{W_{K}^{T}\chi_{a,i}}}, \end{array}$$

where *y*_*a*,*i*_ is the label of image *χ*_*a*,*i*_, *P* is the number of person identities, and *K* is the number of people with this identity. In addition, the batch hard triplet loss is defined in the following equation:

(6) $$\begin{array}{c} L_{\text{BH}}=\sum_{i=1}^{P}\sum_{a=1}^{K}\left[m+\overset{\begin{array}{cc} \text{hardest} & \text{positive} \end{array}}{\overset{︷}{\underset{p=1...K}{\max}E\left(X_{a}^{i},X_{p}^{j}\right)}}-\overset{\begin{array}{cc} \text{hardest} & \text{negative} \end{array}}{\overset{︷}{\underset{\begin{array}{c} j=1...p\\ n=1...K \end{array}}{\min}E\left(X_{a}^{i},X_{n}^{j}\right)}}\right], \end{array}$$

where *X*_*a*_^*i*^ is the anchor sample, *X*_*p*_^*j*^ is the hard positive sample of *X*_*a*_^*i*^, and *X*_*n*_^*j*^ is the hard negative sample of *X*_*a*_^*i*^. The overall process of our proposed method is described in Algorithm 1.

## 4. Experiment

### 4.1. Dataset

Experiments were conducted on the Market-1501 dataset and DukeMTMC-reID dataset to evaluate the effectiveness of the SMCC method. The Market-1501 [24] dataset is a popular dataset for person re-ID, and it contains 32668 people images with 1501 identities. The training set consists of 12,936 images with 751 identities, the test set consists of 19,732 images of 750 identities, and the query set consists of 3368 images. The DukeMTMC-reID [25, 26] dataset consists of 16,522 training set images with 702 identities captured by 8 different cameras, 2228 query set images of 702 identities, and 17,661 gallery images.

### 4.2. Implementation Details

We initialize the parameters of ResNet-50 [59] on ImageNet [60] and use it as the backbone of the model. We resize the input image to 256 × 128 and enhance the diversity of the samples by horizontal flipping, random cutting, and erasing. To obtain a model adapted to the source domain, we use SPGAN [51] to transfer the style of the images in the source domain and generate a style transfer dataset to pretrain the model. After that, we implement the HDBSCAN method to cluster the samples and generate pseudolabels and pseudolabels' confidence levels according to the IDC value of each sample within the cluster. In the process of clustering, space transformation is performed to establish the minimum spanning tree. In the established HDBSCAN tree, the distance of samples within the cluster is sorted, and the weight of sample points is assigned according to the ranking. The weight of credibility is used to recalculate the distance of mutual reachable between samples, which range from 0.1 to 0.9. After that, the reachable distance between samples is sorted, the cluster hierarchy is compressed, and the clustering results are finally extracted. The unclustered outliers are discarded at the end of the clustering process. We select the first eight samples from each cluster according to the IDC ranking list. The threshold of the KCP measurement is set to 0.7. We regard sample points with high IDCs that are greater than the KCP threshold as credible samples. We generate a new credible dataset containing credible samples to fine-tune the model. The loss function of SMCC consists of the hard batch triplet loss [57]. We set the SGD optimizer's initial learning rate to 6 × 10^−5^ and its momentum to 0.9. The whole training process has 30 iterations, and each iteration contains 80 epochs. When the loss function converges, we test the model on gallery set and get the highest mAP (70.2%) after the 21st iteration on the Market-1501 dataset. And, we test the model on gallery set and get the highest mAP (63.4%) after the 23rd iteration on the DukeMTMC-reID dataset.

### 4.3. Ablation Studies

To verify the effectiveness of each criterion of our proposed SMCC method, we conduct extensive experiments on the Market-1501 dataset and DukeMTMC-reID dataset. We use the source domain images after style transfer to pretrain the model, cluster the model with the HDBSCAN method, and use this model as the baseline for ablation studies to explore the improvements in model performance yielded by the IDC and KCP criteria. The comparison results are shown in Tables 1 and 2. In Table 1, the DukeMTMC-reID dataset is the source domain and the Market-1501 dataset is the target domain. In Table 2, the Market-1501 dataset is the source domain and the DukeMTMC-reID dataset is the target domain.

Tables 1 and 2 show that the supervised model is trained and tested on the same dataset, so the Rank-1 and mAP on the Market-1501 dataset reach 92.0% and 80.9%, respectively. However, when we directly apply the model trained in the source domain to the unlabelled Market-1501 dataset, the Rank-1 and mAP are significantly reduced to 48.7% and 25.1%, respectively, due to the existence of domain shift. This is also one of the reasons why person re-ID in the closed world cannot be effectively implemented. Rather than executing a direct transfer, we use SPGAN to transfer the style of the source domain images to the labelled images, whose style is similar to the style of the target domain, and use them as pretraining samples. After that, we fine-tune the model with the pseudolabels obtained by the HDBSCAN method. The performance obtained by the baseline model is better than that obtained by direct transfer.

Next, we introduce the IDC measurement criteria with respect to the baseline to select credible samples for training the model. After the introduction of the IDC, the Rank-1 and mAP of the model on the DukeMTMC-reID dataset are improved by 5.3% and 4.6%, respectively. Similarly, after the introduction of the IDC, the model's Rank-1 and mAP on the Market-1501 dataset improve by 3.6% and 3.7%, respectively. The experimental results show that the IDC can select more credible samples for training. Starting from the baseline, we separately introduce the KCP measurement criterion as the method of credible sample selection. After introducing the KCP, the Rank-1 and mAP of the model on the DukeMTMC-reID dataset are improved by 4.1% and 3.0%, respectively. Similarly, after the introduction of the KCP, the Rank-1 and mAP of the model on the Market-1501 dataset are improved by 2.7% and 2.8%, respectively. This shows that the KCP can improve the performance of the model from the perspective of the spatial distribution of the *K*-reciprocal nearest neighbour samples. We set different KCP thresholds for the baseline on Market-1501 and DukeMTMC-reID to determine an optimal threshold. As shown in Figure 3, when the KCP threshold is 0.7, the model performs best. When the KCP threshold is low, the noisy samples are still regarded as credible samples for optimizing the model. Although a small portion of the falsely labelled samples are filtered out, the performance improvement achieved by the model is relatively weak. With the increase in the KCP threshold, the CMC and accuracy score of the model reach their maximum values. When the KCP threshold is greater than 0.7, the number of credible samples decreases due to the high threshold, which inevitably leads to the overfitting problem, and the robustness of the model is gradually reduced. In addition, we introduce the IDC and KCP to the baseline at the same time; hence, the Rank-1 and mAP scores increase by 8.7% and 11.9% on DukeMTMC-reID and 6.5% and 8.0% on Market-1501, respectively. Although the IDC and KCP are two different confidence measurement criteria, most of the credible samples selected by these two methods meet these two conditions simultaneously. We also evaluate different clustering methods. The performance of these clustering methods under the same network structure is shown in Tables 3 and 4.

As seen from Tables 3 and 4, the *K*-means algorithm, as one of the traditional partition clustering methods, has performance that is heavily dependent on the selection of the initial points and the value of *K*, and the clustering results are easily affected by random initial points; thus, the algorithm is not sufficiently stable. It obtains an mAP of 63.1% and a Rank-1 of 81.3% on the Market-1501 dataset. The CURE [61] hierarchical clustering algorithm, despite its great performance in complex spaces, is strict in terms of its parameter settings and is sensitive to spatial data density. It yields a 5.3% map improvement and 3.6% Rank-1 improvement compared to the *K*-means algorithm. Additionally, as a hierarchical clustering algorithm, the BIRCH [62] algorithm can quickly obtain clustering results by constructing a clustering feature tree and clustering the nodes of the clustering feature tree, but the clustering results are somewhat different from the actual feature distribution. In contrast, the DBSCAN [63] algorithm is able to resist noise and cope with different cluster structures. However, our SMCC method using HDBSCAN is superior to other clustering algorithms. On the DukeMTMC-reID dataset, we obtain 63.4% mAP and 79.1% Rank-1, which are 1.7% and 1.4% higher than those of CURE and 1.3% and 1.1% higher than those of DBSCAN, respectively. Our method can select credible pseudolabels from each cluster for model training after obtaining clustering results, avoid the damage caused by outliers to the stability of the model, and exhibit better performance under different densities.

The above experimental results prove that the SMCC method improves the model performance by selecting samples. In the feature space, based on the positions of the samples, it not only avoids the abnormal selection of sample points, but the KCP criterion used to simultaneously explore the *K*-reciprocal nearest neighbour also enables the proposed method to avoid the selection to samples far from the median centre which may cause misleading results in the training process. Together, these two criteria can promote each other and better cope with the challenge of excessive outliers with respect to the stability of the model during training.

### 4.4. Comparison with the State-of-the-Art Approach

We compare the proposed SMCC method with the state-of-the-art UDA person re-ID method. The experimental training set is DukeMTMC-reID, the test set is Market-1501, and vice versa. The comparison results are shown in Tables 5 and 6. The experimental results demonstrate the efficiency of our SMCC method.

Tables 5 and 6 show that although PTGAN [50], SPGAN [51], HHL [15], and CR-GAN [52] can improve the model performance, CR-GAN outperforms other style transfer methods. Although it improves the performance of the model, due to the lack of utilization of unlabelled target domain data, their performance is slightly inferior to that of the UDA person re-ID method which generates false labels by clustering. We also compare the EANet method [64], which aligns the body's key points, and our method obtains mAP and Rank-1 scores that are 18.6% and 8.5% higher than those of EANet, respectively. CAMEL [16], a method that attempts to align image feature space information under different views, also fails to fully explore label information. In addition, compared with the UDA re-ID method which generates pseudolabels by clustering, the UDAP [7] method performs clustering on the target domain and achieves better results than the style transfer method. Regarding the clustering-based methods, the PAUL [54] and SSG [55] approaches, which combine global features and local features, cannot ensure the correctness of the pseudolabels generated by clustering, and the model performance easily decreases with incorrect labels. Our method outperforms the above methods by selecting credible samples to reduce the misleading label noise of the model. With the continuous optimization of the feature spatial distribution, an increasing number of credible samples are added into the training process, which effectively reduces the influence of overfitting. Compared with the semisupervised person re-ID method SSG++ [55], our method also has some advantages. AD-Cluster [46] adopts a GAN to enhance the image diversity under the same camera settings and uses adversarial learning to optimize the resultant model. Our SMCC method obtains a Rank-1 score that is 0.2% less than the Rank-1 score of AD-cluster on the Market-1501 dataset, but the other evaluation indexes are the best among all methods. The SMCC method can fully explore the feature space distribution of the target domain and select credible sample points from the current cluster and adjacent points by the IDC and KCP, which can reduce the impact of label noise on the model during the initial stage of training and ultimately improve the performance of the model. The experimental results verify the effectiveness of our proposed SMCC method.

## 5. Conclusions

In this paper, stable median centre clustering for the unsupervised domain adaptation person re-ID method is proposed. The credible samples near the median centres of clusters are selected by the intracluster distance confidence degrees. We also use the *K*-reciprocal neighbour cluster proportion of the sample to ensure that the selected samples are relatively concentrated in the spatial distribution and reduce the influence of outliers with label noise on model training. Furthermore, we propose a new method to measure intercluster sample distances according to the intracluster distance confidence ranking list; this method assigns different weights to different samples, increases the contributions of credible samples to the distance calculation to reduce the impact of label noise, and pays more attention to the contribution of stable samples to training, while ensuring the calculation of all sample points. This forces the model to fully explore the potential similarities among credible samples. The experimental results demonstrate the effectiveness of our SMCC method compared to that of the state-of-the-art methods.

## Figures and Tables

**Figure 1:** Iterative adjustment process for credible sample selection. As the number of iterations increases, the number of credible samples gradually increases. The distances between samples belonging to the same cluster in the feature space are smaller, and the distances between samples belonging to different clusters are larger. Finally, the credible samples are used for training to prevent the influence of label noise on the model.

**Figure 2:** Overview of the SMCC method. First, we use SPGAN [51] to transfer the image style of the source domain to images with styles similar to the target domain style while preserving the person identity, and we pretrain the CNN model on these data. After that, HDBSCAN [56] is performed on the feature vectors obtained by feature extraction based on the target domain data of the CNN model. Due to the noise in the labels, we select credible samples according to the IDC and KCP of the samples to optimize the CNN model by the batch hard triple loss [57] and softmax cross-entropy loss.

**Figure 3:** The CMC and accuracy score of the model under different KCP thresholds. (a) Market-1051 dataset. (b) DukeMTMC-reID dataset.

**Algorithm 1:** Stable median centre clustering.

**Table 1:** Ablation studies regarding SMCC on Market-1501. Supervised model: the re-ID model for which training and testing are conducted in the target domain. Direct transfer: the re-ID model pretrained in the source domain is directly transferred to the target domain. Baseline: the re-ID model uses SPGAN to conduct style transfer on the images for pretraining and then performs the HDBSCAN method. IDC : the intracluster distance confidence. KCP : the *K*-reciprocal nearest neighbour cluster proportion.

Method	DukeMTMC-reID⟶Market-1501			
	Rank-1	Rank-5	Rank-10	mAP
Supervised model	92.0	97.4	98.4	80.9
Direct transfer	48.7	69.5	76.9	25.1
Baseline	77.8	85.7	89.1	58.3
Baseline + IDC	83.1	92.2	95.5	62.9
Baseline + KCP	81.9	91.8	93.9	61.3
Baseline + IDC + KCP	86.5	94.6	96.7	70.2

**Table 2:** Ablation studies regarding SMCC on DukeMTMC-reID.

Method	Market-1501⟶DukeMTMC-reID			
	Rank-1	Rank-5	Rank-10	mAP
Supervised model	82.6	92.1	94.6	70.2
Direct transfer	29.7	44.1	50.4	16.2
Baseline	72.6	82.0	85.3	55.4
Baseline + IDC	76.2	84.9	87.7	59.1
Baseline + KCP	75.3	83.5	87.0	58.2
Baseline + IDC + KCP	79.1	86.8	89.1	63.4

**Table 3:** Performance of different clustering algorithms on the Market1501 dataset.

Clustering method	DukeMTMC-reID⟶Market-1501			
	mAP	Rank-1	Rank-5	Rank-10
*K*-means	63.1	81.3	88.0	90.9
CURE [61]	68.4	84.9	93.1	94.7
BRICH [62]	68.9	84.0	92.4	93.1
DBSCAN [63]	69.5	85.6	93.3	95.6
Ours	70.2	86.5	94.6	96.7

**Table 4:** Performance of different clustering algorithms on the DukeMTMC-reID dataset.

Clustering method	Market-1501⟶DukeMTMC-reID			
	mAP	Rank-1	Rank-5	Rank-10
*K*-means	58.4	74.1	82.3	84.9
CURE [61]	61.7	77.6	84.4	87.2
BRICH [62]	61.4	77.3	84.0	86.6
DBSCAN [63]	62.1	78.0	85.2	88.1
Ours	63.4	79.1	86.8	89.1

**Table 5:** The comparison of our proposed SMCC method with the state-of-the-art method on Market-1501.

Method	DukeMTMC-reID⟶Market-1501			
	mAP	Rank-1	Rank-5	Rank-10
PTGAN [50]	—	38.6	—	66.1
SPGAN [51]	22.8	51.5	70.1	76.8
HHL [15]	31.4	62.2	78.8	84.0
CR-GAN [52]	54.0	77.7	89.7	92.7
EANet [64]	51.6	78.0	—	—
CAMEL [16]	26.3	54.5	—	—
PAUL [54]	40.1	68.5	82.4	87.4
UDAP [7]	53.7	75.8	89.5	93.2
PAST [20]	54.6	78.4	—	—
SSG [55]	58.3	80.0	90.0	92.4
AD-cluster [46]	68.3	86.7	94.4	96.5
SSG++ [55]	68.7	86.2	94.6	96.5
Ours	70.2	86.5	94.6	96.7

**Table 6:** The comparison of our proposed SMCC method with the state-of-the-art method on DukeMTMC-reID.

Method	Market-1501⟶DukeMTMC-reID			
	mAP	Rank-1	Rank-5	Rank-10
PTGAN [50]	—	27.4	—	50.7
SPGAN [51]	22.3	41.1	56.6	63.0
HHL [15]	27.2	46.9	61.0	66.7
CR-GAN [52]	48.6	68.9	80.2	84.7
EANet [64]	48.0	78.0	—	—
CAMEL [16]	—	—	—	—
PAUL [54]	53.2	72.0	82.7	86.0
UDAP [7]	49.0	68.4	80.1	83.5
PAST [20]	54.3	72.4	—	—
SSG [55]	53.4	73.0	80.6	83.2
AD-cluster [46]	54.1	72.6	82.5	85.5
SSG++ [55]	60.3	76.0	85.8	89.3
Ours	63.4	79.1	86.8	89.1

## Data Availability

The data used to support the findings of the study are available from the corresponding author upon request.
